# Comparative Study of Artificial Intelligence Techniques for the Diagnosis of Chronic Nerve Diseases

This article has been retracted.

**DOI:** 10.1155/2022/3522510

**Published:** 2022-01-13

**Authors:** Saud Aljaloud, Jalawi Alshudukhi, Khalid Twarish Alhamazani, Assaye Belay

**Affiliations:** ^1^College of Computer Science and Engineering, Department of Computer Science, University of Ha'il, Saudi Arabia; ^2^Department of Statistics, Mizan-Tepi University, Ethiopia

## Abstract

Farming is essential to the long-term viability of any economy. It differs in each country, but it is essential for long-term economic success. Only a few of the agricultural industry's issues include a lack of suitable irrigation systems, weeds, and plant monitoring concerns as a consequence of efficient management in distinct open and closed zones for crop and plant treatment. The objective of this work is to carry out a study on the use of artificial intelligence and computer vision methods for diagnosis of diseases in agro sectors in the context of agribusiness, demonstrating the feasibility of using these techniques as tools to support automation and obtain productivity gains in this sector. During the literary analysis, it was determined that technology could improve efficiency, hence decreasing these types of concerns. Given the consequences of a wrong diagnosis, diagnosis is work that requires a high level of precision. Fuzzy cognitive maps were shown to be the most efficient method of utilizing bibliographically reviewed preferences, which led to the consideration of neural networks as a second option because this technique is the most robust in terms of the qualifying criteria of the data stored in databases.

## 1. Introduction

### 1.1. Artificial Intelligence and Phytosanitary Diagnostics

Diagnosis, in humans, animals, and plants, is an activity carried out by specialists with expertise in the field in which the diagnosis process is carried out. Artificial intelligence tries to emulate the natural ability that human beings have to make decisions of any archetype, simulating in their way of learning how that instruction is based on reaching decision-making [1]. The agricultural sector is one of the essential sectors globally speaking; however, it has been the victim of losses due to diseases, taking into consideration that people with problems of poverty live in these areas, which makes this group of farmers very vulnerable being interrupted in the supply of food products derived from pathogens [2, 3]. For this purpose, various artificial intelligence techniques have been used, including neural networks, expert systems (already mentioned above), data mining, and intelligent agents. In recent decades, some efforts have been made to apply predictive analysis to health systems and to activate machine learning systems that facilitate the diagnosis of diseases [4]. For the diagnosis of diseases in agriculture, the quick and easy integration of the contents that can replace the old diagnosis is a primary cause, being that the diagnosis is a highly complex process, which is not accurate and cannot be carried out to term without previously considering other alternatives, due to the uncertainty present in the procedure [5, 6]. As a result of this great uncertainty, the determinations that the different specialists have adopted in each stage of the diagnostic procedure are not always the same, since each specific incident entails a different decision procedure for each specialist, although this is trying the assessment of the same type of condition. There are ways to identify any plant's conditions, such as examining plant tissues in an equipped laboratory or the presence of a specialist agronomist at the planting site; in either case, the problem is the time it takes to get the results [2]. Among the techniques that have been used most frequently for the recognition of diseases, the following stand out: fuzzy logic (diagnosis based on classification), expert systems (based on rules, probabilities, based on cases), neural networks (diagnosis based on training and recognition), and applied data mining (diagnosis based on pattern recognition) [1]. These techniques have substantial potential in artificial intelligence in agriculture.

Again, the contrast research is an important component in determining which artificial intelligence approach is best suited to diagnosing agricultural illnesses. The examination of fuzzy cognitive maps is used to determine which artificial intelligence approach is most suited to illness diagnosis. Fuzzy cognitive maps have become one of the most widely used and researched AI approaches in recent years. The need to construct causality models that are more realistic, as well as the necessity for accuracy and interpretability, has prompted an upsurge in research into this sort of mathematical representation [8]. This study provides an overview of artificial intelligence-based diagnostic reasoning methodologies (AI). It provides an outline of the history of various techniques. Due to the limitations of existing approaches, a group of researchers resorted to experienced physicians for profound insights into the underlying nature of clinical situation, as well as artificial intelligence to put these insights into practical programs. In addition, as understanding of the information processing qualities of computer models of cognitive processes improves, efficient data structures and algorithms are often designed to execute the same behavior on computers that bear little, if any, resemblance to the original models. This chapter discusses the development of some of these models as well as its applications in the field of general medical diagnosis. It examines the evolution of computational techniques in the area of medical diagnosis. The chapter also looks at a range of systems that are becoming more capable and complicated, with an emphasis on the link among representation of knowledge and logical thinking, as well as how our insight into the nature of diagnosing expertise has changed over time. It also offers a description of a sequential diagnostic procedure Bayesian belief probability theory [7].

These provide a potent technique for modeling and predicting complex systems that is extremely multivariable and interpretable. MCD's core principle is to regulate the object of research by breaking it into primary parts and then describing the dynamics of internal interactions between these elements [9].

## 2. Materials and Methods or Methodology

The research adopted a quantitative approach. Decision theory was used, beginning with the identification and definition of the problem and ending with the choice of one or more possibilities, which involves a decision-making exercise, a procedure that is based on five essential stages. Decision-making, in the present work, focuses on the search for the best technique commonly used to diagnose diseases in agriculture. The process begins with the identification and definition of the problem and ends with the selection of one or more variants, which implies the act of making a decision.

Based on the information previously registered in databases, five phases have been determined to decide on the best artificial intelligence technique, which is used regularly in the diagnosis of agricultural diseases. The initial stages of the decision-making procedure consist of articulating the problem and the last two in analyzing it [10]. The stages for the conclusion of an incident through decision-making are presented (Figure 1):

The research stage of the decision-making process can take two main formats: qualitative and quantitative. Qualitative analysis is based on the reasoning and practice of the entity that made the decision; it includes your intuitive impression of the problem. Using the quantitative approach, the researcher focuses on the data or factors that relate to the incidence and leads to the development of exact science expressions that describe the problem's purposes, limitations, and interactions [11]. Then, using quantitative methods, it is possible to offer a suggestion based on the quantitative components of the problem.

In this sense, we have to know the best way to evaluate to determine which artificial intelligence technique is best adapted to the diagnosis of diseases in agriculture, considering the peculiarities of each technique:

1. The first stage (A): it is carried out continuously on the advantages of AI practices used in diagnoses, in which plant pathology professionals have an expert role in obtaining knowledge
2. The second stage (B): the evaluation of AI techniques is carried out, presenting case studies to make comparisons, the criteria of experts prevail, and the comparison with data stored in databases
3. Third stage (C): agronomists or phytopathologists (experts) can raise and solve problems related to their field and imply the knowledge built during the determined time of the presence of disease symptoms

Legend:

1. General principle (based on)
2. A specific branch of artificial intelligence
3. Classification within the branch of artificial intelligence
4. Application

To select the technique that best fits the process of diagnosing diseases in agriculture, it is recommended to consider each technique's principle.

1. (1—expert system) based on obtaining knowledge
2. (2—neural networks) based on training and classification
3. (3—intelligent agents) based on the interrelation with the environment

Establish the best way to evaluate the diagnoses with the cases previously stored in the databases in agriculture. When establishing the fuzzy cognitive maps since it forms globalization of the cognitive maps, both are directed graphs, whose vertices represent concepts and their edges represent causal relationships between these concepts [12]. The difference is in the values assigned to the edges that signify the degree of relationship between the vertices. In cognitive maps, these values are −1, 1, which suppose an inverted or direct correlation between the concepts. In comparison, fuzzy cognitive maps take values in the range [−1, 1], where a scale is included between the differences of the concepts [13].

### 2.1. Steps to Follow to Apply the Fuzzy Cognitive Map Method

These are directed graphs that use vertices to represent the concepts or variables in scope. At the same time, the edges indicate positive, negative, or null causality relationships between the terms represented by the vertices. Fuzzy cognitive maps (FCMs) extend cognitive maps to the fuzzy domain in the interval [−1, 1] to determine the strength in causal relationships [14]. FCM refines cognitive maps, which describe joint strength through fuzzy data in the interval [−1, 1] [2].

Cognitive maps help us to show the causal interrelationships between the variables, where each edge is related to a weight value in the set, being 0 the one that indicates that there is no causal relationship between the variables, -1 means that the relationship of causality is inverse (if one variable increases and the other decreases), and one means that there is a direct causality relationship (both variables are increasing or both are decreasing) [15]. These factors do not cover the uncertainty in these causal relationships, which causes fuzzy cognitive maps to emerge. It is possible to introduce a classification in the previous set of weights defined in the continuous interval [−1, 1].

There are three classes of possible causal relationships between concepts in FCMs:

1. Causality is positive (*W*_*ij*_ > 0): there is a directly proportional causality between the concepts *C*_*i*_ and *C*_*j*_, that is, the increase (decrease) in the value of *C*_*i*_ leads to the increase (decrease) of the value of *C*_*j*_
2. Causality is negative (*W*_*ij*_ > 0): there is an inversely proportional causality value of *C*_*i*_ and *C*_*i*_, that is, the increase (decrease) of the value of *C*_*i*_ leads to the decrease (increase) in the value of *C*_*i*_
3. The nonexistence of relationships (*W*_*ij*_ > 0): this indicates the nonexistence of a causal correlation between *C*_*i*_ and *C*_*j*_

We propose in this study, based on cognitive maps for decision-making, the following algorithm:

(1) The selection of the most relevant causes
(2) Once the most relevant causes have been selected, the causality between them will be modeled with the help of a fuzzy cognitive map
(3) Static analysis [15]: the following measures are scored for the absolute results of the adjacent matrix:
  - Outdegree, which is identified with od (vi), is the sum for each row of the absolute values of a variable in the adjacent fuzzy matrix. It is a measure of the cumulative strength of the existing relationships of the variable
  - Indegree, which is identified by id (vi), is the sum of each column of the absolute results of one of the variables of the adjacent fuzzy matrix. This measures the cumulative input force of the variable
  - The centrality or the degree of the totality of the variable is the sum of od (vi), where id (vi) is as follows: td (vi) = od (vi) + id (vi)

In the end, these variables can be classified according to the following criteria, according to authors [16]:

- Transmission variables are those that contain *e*
- The receiving variables are those with and
- Common or ordinary variables comply with and

They are managed in ascending order according to the degree of centrality.

Due to the significant utility of fuzzy cognitive maps, they have been recognized to model various scenarios. This being the case, we were able to find extensions based on intervals, intuitionist fuzzy logic [16], among other extensions.

A diffuse cognitive map can be represented by a digraph (Figure 2) using which these nodes manage to represent the criteria, and then, the arcs show us a causal link.

When a group of experts (*κ*) participates, the adjacent matrix can be formulated using an aggregation operator, such as the arithmetic mean. The most straightforward tactic is to find the mean on each connection for each proficient.

For (*κ*) individuals, the final adjacent matrix of the FCM (*E*) is obtained as [17]

(1) $$\begin{array}{c} E=\frac{\left(E_{1}+E_{2}+\cdots +E_{k}\right)}{k}. \end{array}$$

This ease of aggregation allows us to create collective mental models with relative simplicity. This method allows us schemes that are as close to reality as possible to represent knowledge. Among the factors that facilitate an interpretation of knowledge as authentic as possible is the opportunity to represent the cycles, vagueness, and ambiguity present and also great ease of use for obtaining knowledge by farmers.

## 3. Results and Discussion

To obtain the results of the current problem, it is necessary to develop the following model, taking into account each criterion that has been frequently used for the diagnosis of diseases in agriculture through bibliographic review (Figure 3).

The following evaluation criteria were considered in the model in each of the artificial intelligence techniques raised above:

- Accuracy
- Learning capacity
- Interpretability
- Adaptability
- Efficiency

The suitability of the method is the factor that evaluates the three artificial intelligence techniques to be able to choose the best of these.

We will start with the description in the following tables of the artificial intelligence techniques and their corresponding criteria, to later represent them graphically by means of a hyperbolic tangent and then present the result of the method used by means of fuzzy cognitive maps.

Next, in Table 1, we locate the values of the criteria of the expert system technique.

It is graphed showing us the result of 0.89 in the criterion of suitability of the method.

Table 2 refers to the values of the neural network technique criteria.

It is graphed showing us the result of 0.98 under the criterion of appropriateness of the method in the neural network technique.

Table 2 refers to the values of the criteria of the multiagent system technique.

It is graphed showing us the result of 0.82 in the criterion of suitability of the method of the multiagent system technique.

Finally, we will show in Table 3 the measures of centrality based on the absolute value of the adjacency matrix where the result of the centrality td (vi) = od (vi) + id (vi) is the total sum of the values of the indegree and outdegree criteria.

According to the analysis carried out and according to the results that are displayed in the total matrix of adjacent results, the value of the most qualified criterion is the suitability of the method, achieving the artificial intelligence technique with the highest value neural networks, giving as a result, neural network is the technique that best adjusts for the diagnosis of diseases in agriculture, taking into consideration the criteria with which it has been evaluated in this study using a bibliographic review and applying fuzzy cognitive maps.

The result is verified when relating and putting into practice diagnostics in agriculture based on artificial intelligence techniques, particularly using data stored in databases. In this sense, it stands out that neural network is one of the most powerful artificial intelligence tools. They have the provision of learning a group of matrices and structural weighting data to represent the learning of the different models [18].

Neural networks are adjusted for the diagnosis of diseases in agriculture since they are composed of numerous processing units, simulating the brain's functionality and the way of performing functions as a living being [19]. Neural networks have been frequently applied in various phytosanitary diagnosis applications, obtaining very favorable results and with a higher degree of certainty than other artificial intelligence techniques, which they provide in phytosanitary diagnoses [20].

## 4. Conclusions

The various artificial intelligence tools were analyzed for the detection of phytosanitary diseases in agriculture, each of which has been of great importance; this process, which has been supported by artificial intelligence throughout history, has been able to represent precise results by using them, specifically in the area of agriculture, different disease diagnoses have been developed [21, 22]. In this study carried out, the following artificial intelligence techniques, neural networks, expert systems, and multivalent systems, were bibliographically verified, considering the principle of each technique, based on fuzzy cognitive maps for decision-making in algorithms. Each of the characteristics of the artificial intelligence techniques was evaluated, thus obtaining the most efficient through the instrumentalization of the bibliographically reviewed preferences through fuzzy cognitive maps, which led to consider the second alternative, neural networks, since this technique is the most robust in terms of the qualifying criteria of the data stored in databases.

## Figures and Tables

**Figure 1:** Phases for solving a problem through decision-making.

**Figure 2:** Fuzzy cognitive map.

**Figure 3:** Diffuse cognitive map model.

**Table 1:** Evaluation table of expert system criteria.

Criteria	+/−
Learning capacity	0.51
Interpretability	0.78
Adaptability	0.18
Precision	0.77
Efficiency	0.33
Appropriateness of the method	

**Table 2:** Multiagent system criterion evaluation table.

Criteria	+/−
Learning ability	1.01
Interpretability	0.26
Adaptability	0.97
Accuracy	1.02
Efficiency	0.90
Appropriateness of the method	

**Table 3:** Matrix table of adjacent results.

Criteria	Indegree	Outdegree	Centrality
Learning capacity	0.47	1.25	1.72
Interpretability	0.00	0.89	0.89
Adaptability	0.00	0.92	0.92
Precision	0.69	0.59	1.28
Efficiency	0.00	0.31	0.31
Appropriateness of the method	2.80	0.00	2.80

## Data Availability

The data underlying the results presented in the study are available within the manuscript.
